# Dark-Lumen Magnetic Resonance Image Based on Artificial Intelligence Algorithm in Differential Diagnosis of Colon Cancer

**DOI:** 10.1155/2022/4217573

**Published:** 2022-03-27

**Authors:** Yujie Fang, Ting Kang, Yang Yang, Yonghong Zi, Xiong Lu

**Affiliations:** ^1^Department of Geriatric Gastroenterology, Xi'an No. 1 Hospital, Xi'an 710002, Shaanxi, China; ^2^Department of Oncology, Affiliated Hospital of Yan'an University, Yan'an 716000, Shaanxi, China; ^3^Department of General Surgery, Baoji People's Hospital, Baoji 721000, Shaanxi, China; ^4^Department of Gastroenterology, Affiliated Hospital of Yan'an University, Yan'an 716000, Shaanxi, China

## Abstract

This research was aimed *o* investigate the application value and diagnostic effect of dark-lumen magnetic resonance imaging (dark-lumen MRI) based on artificial intelligence algorithm on colon cancer. A total of 98 patients with ulcerated colon cancer were selected as the study subjects. All patients underwent colonic endoscopy. The patients were divided into algorithm group (artificial intelligence algorithm processing image group) and control group (conventional method processing image group) according to different dark-lumen MRI processing methods. The detection efficiency of colon cancer was compared between the two groups. It showed that the diagnostic effect of dark-lumen MRI based on artificial intelligence algorithm was significant. The apparent diffusion coefficient (ADC) in the control group was 0.92 ± 0.14 mm^2^/*s* (minimum: 0.74, maximum: 1.30), ADC in the algorithm group was 1.55 ± 0.31 mm^2^/*s* (minimum: 1.22, maximum: 2.42). The ADC of patients in algorithm group was significantly higher than that of patients in control group, with statistical difference (*t* = 7.827, *P* *<* 0.001). The correct number of cases was 46 and the diagnostic error number was 3 in algorithm group, with accuracy of 93%. The correct number of cases was 41 and the diagnostic error number was 8 in control group, with accuracy of 83%. In comparison, the correct rate was 10% higher in algorithm group, indicating that the diagnostic effect was better in algorithm group. The mean value of invasion depth was 10.42 in the algorithm group and 5.27 in the control group, indicating that the algorithm group was more accurate in the judgment of invasion depth, had a good prospect of clinical application, and had guiding significance for the diagnosis of colon cancer.

## 1. Introduction

With the change of people's living and eating habits, the incidence rate of colon cancer has been greatly increased [1]. Statistical data show that colon cancer ranks second in the incidence of cancer [2]. The most common type of colon cancer is ulcerative colon cancer, which is usually examined by imaging [3]. Studies have shown that the course and development of ulcerative colitis is important for cancer detection [4]. However, conventional examination methods are often limited by the narrow intestinal tract caused by colon cancer [5, 6]. Colonoscopy can detect potential bleeding in colon, for colon polyps and colon cancer screening, but less experienced experts, and the requirements of colonoscopy are strict [7, 8]. In addition, colonoscopy cannot evaluate the degree and nature of lesions, which will reduce the detection rate of colon cancer [9, 10], so it is not easy to popularize. The sensitivity and specificity of ultrasonography in the diagnosis of colon cancer are 67 %–86% and 79 %–87%, respectively. In addition, ultrasound is also affected by many factors, such as the operator's ability.

It was demonstrated that magnetic resonance imaging (MRI) examination is the most accurate image examination method for rectal cancer, and the application of abdominal coil completely shows the invasion of extraintestinal lesions with advantages compared with t3 and t4 tumors [11]. In MRI, diffusion-weighted imaging (DWI) and functional MRI assess the effectiveness of chemoradiotherapy and play an important role in detecting tumor recurrence [12]. Dark-lumen magnetic resonance colonography (Dark-lumen MRC) refers to an MRI technique for the detection of the large intestine and is the examination of injecting an appropriate amount of hot water into the anus. Combined with artificial intelligence image enhancement technology, small ulcers or polyps of colon cancer in ulcerative colorectal lesions can be clearly observed [13]. Bergman dictionary learning algorithm has remarkable effect in improving the quality of MRI images, and has been widely studied [14]. However, there are relatively few studies on its application in the treatment of colon cancer. Zlochower et al. (2020) [15] reported a diagnostic sensitivity of 50% and 84.6% for dark-lumen MRC above 10 mm for colonic lesions of 6 mm - 9 mm, respectively. However, the relatively high cost of MRC is somewhat difficult to use widely in clinics. 98 patients with ulcerative type colon cancer (UTCC) were selected as the study subjects for colon cancer examination in order to provide a reference for improving the efficiency of early diagnosis of colon cancer.

## 2. Methods

### 2.1. Subjects

A total of 98 patients with UTCC were selected as the study subjects. All patients underwent colonic endoscopy. The patients were divided into algorithm group (artificial intelligence algorithm processing image group) and control group (conventional method processing image group) according to different dark-lumen MRI processing methods. The detection efficiency of colon cancer was compared between the two groups. This study had been approved by the ethics committee of hospital, and the patients and their family members signed the informed consent form.

Inclusion criteria: (1) patients have clinical symptoms of localized or diffuse circular thickening of the intestinal wall. (2) No other sudden diseases (such as hypertension, heart disease, diabetes). (3) No sensitive symptoms of anisodamine. (4) Patients with nonrejection of lumen MRI.

Exclusion criteria: (1) patients who did not sign the informed consent form. (2) Patients with other cancers. (3) Patients under 18 years of age. (4) Patients with other inflammatory diseases. (5) Patients with systemic diseases such as systemic lupus erythematosus. (6) Patients using nonsteroidal anti-inflammatory drugs, glucocorticoids, and immunosuppressive agents.

### 2.2. Bergman Iterative Algorithm for Artificial Intelligence

The problem that the Bergman algorithm first to solve is as follows.

(1) $$\begin{array}{c} \;\min_{u}J\left(u\right),\\ \text{s}.\text{t}.G\left(u\right)=0. \end{array}$$

The equation for the Bergman distance can be expressed as follows.

(2) $$\begin{array}{c} \;B_{J}^{S}\left(x,y\right)=J\left(x\right)-J\left(y\right)-\langle s,x-y\rangle . \end{array}$$

*J* and *G* are convex functions, *G* is a differentiable function, and *s* is a subgradient presenting in *y*. The excellent feature of the Bergman iterative algorithm is that it can transform the constrained problem into an unconstrained problem.

(3) $$\begin{array}{c} \left\{\begin{array}{c} u^{k+1}=\arg\min_{u}B_{J}^{x^{k}}\left(u,u^{k}\right)+G\left(u\right)\\ s^{k+1}=s^{k}-\nabla G\left(u^{k+1}\right) \end{array}.\right. \end{array}$$

*μ*/2‖*F*_*p*_*u* − *f*^*k*^‖_2_^2^ is used to represent *G*(*u*) in Bergman iteration, and the modified equation is expressed as follows.

(4) $$\begin{array}{c} \left\{\begin{array}{c} u^{k+1}=\arg\min_{u}B_{J}^{x^{k}}\left(u,u^{k}\right)+G\left(u\right)\\ f^{k+1}=f^{k}+f-F_{p}u^{k+1} \end{array}|.\right. \end{array}$$

*u* is taken as the weight coefficient, and ‖*F*_*p*_*u* − *f*^*k*^‖_2_^2^ is taken as the residual term to converge to zero, which is brought into the equation. Finally, the equivalent equation is obtained. The equation can evolve into the following method in practical application.

(5) $$\begin{array}{c} \left\{\begin{array}{c} u^{k+1}=\arg\min_{u}J\left(u\right)+\frac{\mu }{2}{\left\|F_{p}u-f^{k}\right\|}_{2}^{2}\\ f^{k+1}=f^{k}+f-F_{p}u^{k+1} \end{array}|.\right. \end{array}$$

*J*(*u*) denotes the range of the finite difference image, *?* denotes the wavelet transform, *F*_*p*_*u*^*k*+1^ is the regularization weight coefficient, and then the two-step alternating update is solved by the Bergman iteration method to find the optimal mapping relationship.

(6) $$\begin{array}{c} \frac{1}{2}\sum_{i=1}^{M}\sum_{j=1}^{M}{\left(\alpha_{i}-\alpha_{j}\right)}^{2}W_{ij}=Tr\left(\Gamma L\Gamma^{T}\right). \end{array}$$

Combined with the commonly used positioning function, the equation can be obtained.

(7) $$\begin{array}{c} \min_{D,\Gamma }\frac{\lambda }{2}{\left\|X-D\Gamma \right\|}_{F}^{2}+\mu Tr\left(\Gamma L\Gamma^{T}\right)+\sum_{i=1}^{M}{\left\|\alpha_{i}\right\|}_{1},\\ \text{s}.\text{t}.{\left\|d_{j}\right\|}^{2}\leq 1,\;\forall j=1,2,\ldots ,J. \end{array}$$

The objective function is composed of empirical loss term, Laplace regularization term, and sparse penalty term.

*λ* Represents the consistency parameter of the data item, and *?* is the regularization coefficient.

(8) $$\begin{array}{c} \left\{\begin{array}{c} u^{k+1}=\arg\min_{u}\left\{\min_{D,\Gamma }\sum_{i}\left({\left\|\alpha_{l}\right\|}_{1}+\frac{\lambda }{2}{\left\|D\alpha_{l}-R_{i}u\right\|}_{2}^{2}\right)+\frac{\mu }{2}{\left\|F_{p}u-f^{k}\right\|}_{2}^{2}\right\}\\ f^{k+1}=f^{k}+f-F_{p}u^{k+1} \end{array}.\right.. \end{array}$$

The objective function is iterative again, *λ* is the sparse level of the image, *J*=*KM*, *K* can represent the completeness of the database, the spatial constraints of *K* is strengthened, and the problem will also be updated to generate subfunctions.

(9) $$\begin{array}{c} \left(D^{i+1},\alpha_{l}^{i+1},z_{i}^{i+1}\right)=\arg\min_{D,\alpha_{i},z_{i}}\sum_{i}{\left\|\alpha_{l}\right\|}_{1}+\frac{\lambda }{2}{\left\|z_{i}\right\|}_{2}^{2}+\frac{\beta }{2}\left\|z_{i}+D\alpha_{l}-R_{i}u-\frac{y_{l}^{i}}{\beta }\right\|,\\ D^{i+1}=D^{i}+\xi Y^{i+1}{\left(\Gamma^{i+1}\right)}^{T}d_{q}^{i+1}=\frac{d_{q}^{i+1}}{{\left\|d_{q}^{i+1}\right\|}_{2}},\;q=1,2,\ldots ,Q. \end{array}$$

After combining the double-layer Bergman dictionary learning model ‖*α*_*l*_‖_1_+*λ*/2‖*Dα*_*l*_ − *R*_*i*_*u*‖_2_^2^ with the above equation, the solution equation is changed accordingly.

(10) $$\begin{array}{c} \left\{\begin{array}{c} u^{k+1}=\arg\min_{u}\left\{\begin{array}{c} \min_{D,\Gamma }\sum_{i}\left({\left\|\alpha_{l}\right\|}_{1}+\frac{\lambda }{2}{\left\|D\alpha_{l}-R_{i}u\right\|}_{2}^{2}+\mu Tr\left(\Gamma L\Gamma^{T}\right)\right)\\ +\frac{\mu }{2}{\left\|F_{p}u-f^{k}\right\|}_{2}^{2} \end{array}\right\}\\ f^{k+1}=f^{k}+f-F_{p}u^{k+1} \end{array}|.\right. \end{array}$$

To facilitate the solution, *X*=*Ru* is set, and the objective function is transformed into a function with constraints as follows.

(11) $$\begin{array}{c} \min_{D,\Gamma }\frac{\lambda }{2}{\left\|Z\right\|}_{2}^{2}+\mu Tr\left(\Gamma L\Gamma^{T}\right)+{\sum_{i=1}^{M}\left\|\alpha_{i}\right\|}_{1},\\ \text{s}.\text{t}.Z=X-D\Gamma ,{\left\|d_{j}\right\|}^{2}\leq 1,\;\forall j=1,2,\ldots ,J. \end{array}$$

A series of subproblems can be solved by Bergman splitting.

(12) $$\begin{array}{c} \left(D^{k+1},\alpha_{i}^{k+1},z_{i}^{k+1}\right)=\arg\min_{D,\alpha_{i},z_{i}}L_{\beta }\left(D,\alpha_{i},z_{i},y_{i}\right),\\ L_{\beta }\left(D,\alpha_{i},z_{i},y_{i}\right)={\left\|\alpha_{l}\right\|}_{1}+\frac{\lambda }{2}{\left\|z_{i}\right\|}_{2}^{2}+\mu Tr\left(\Gamma L\Gamma^{T}\right)+\frac{\beta }{2}{\left\|z_{i}+D\alpha_{i}-R_{i}u-\frac{y_{l}^{i}}{\beta }\right\|}_{2}^{2}. \end{array}$$

### 2.3. Algorithm Evaluation Indexes

Different sampling rates and sampling trajectories will affect the experimental results, so two-dimensional random sampling mode and different sampling factors are selected for the test. Gaussian white noise is added to the data, the reconstructed image and reconstruction results of the algorithm are compared with the original image. The peak signal-to-noise ratio (PSNR) was used to evaluate the experimental results. All experiments in this study were implemented in MATLAB version 7.11 with a CPU of i7-3632QM and 4 GB of memory for the PC. The equation of PSNR is as follows.

(13) $$\begin{array}{c} PSNR=10\;\log_{10}\left(\frac{255^{2}\times M\times N}{\sum_{w=1}^{M}\sum_{\text{e}=1}^{N}|\text{u}\left(w,e\right)-f{\left(w,e\right)}^{2}}\right). \end{array}$$

### 2.4. Dark-Lumen MRC Inspection

3.0 T magnetic resonance imaging equipment was used for the examination equipment of dark-lumen magnetic resonance, and eight-channel body phased array coil was used for T2-HASTE, DWI, and 3D-DCE-T1-VIBE sequences. The double-barrel dual-channel high-pressure injection contrast medium was 0.2 mL/kg gadopentetate dimeglumine (Gd-DTPA) at an injection rate of 2.0 mL/s. 20 mL normal saline again was injected for contrast medium injection, and the residual drugs in the injection pipeline was washed out.

The low fiber diet was given two days before the MRC examination, 1.5 liters of isotonic electrolyte solution was given orally to the patient before the examination, and the examination could be started when the patient excreted clear water. In patients with tumors that have lesions in the sigmoid or descending colon, bowel cleansing can be performed before examination through low lesion sites. Before the MRC examination, 20 mL of anisodamine needs to be injected within 10–20 minutes. At the same time, the patient performed breathing training. To reduce respiratory motion artifacts during MRC scanning, a respiratory switch was used. Urine pads were required for MRC testing. When 500 ∼ 2,000 mL of warm water was injected, the patient will no longer inject warm water when he/she was uncomfortable. In order to evenly pass the warm water through the intestinal canal, the patient needed to change to lateral decubitus position. At bowel cleansing, MRC was performed with the patient supine.

With the patient in the supine position, a coronal T2-HASTE scan was performed first, with the scan range throughout the colonic lesion, and the images were observed after the scan, and an axial T2-HASTE scan was performed in the affected area with severe disease. Scans were performed axially or in a corneal position, without the need for the patient, *b* at 50 s/mm^2^, 400 s/mm^2^, and 800 s/mm^2^. After scanning, an enhanced 3D-T1-VIBE dynamic examination was performed. After the setup file, a scan program starting 30 seconds after contrast injection was programmed to scan at 30 second intervals. The machine issued a breath-hold command within 10 seconds before each scan cycle with a fixed scan time.

### 2.5. Image Data Measurement Standard

Measurement of intestinal wall thickness: the thick layer near the lesion was selected and the vertical intestinal wall of the membranous side was measured. Region of interest (ROI) selection: the thickest layer of intestinal wall was as close to the thickness of intestinal wall as possible, preventing others. Patients with colon cancer needed to avoid necrotic sites, and the small volume of ROI cannot produce partial volume effect. To reduce measurement error, apparent diffusion coefficient (ADC) and enhanced signal values were measured and averaged over the ROI region. Maximum enhancement value (ME) and relative enhancement ratio (Er) were obtained using the time-signal intensity curve (TIC) given by the workstation. The maximum metric value was the signal intensity when the intestinal enhancement of the affected area reached the peak, and the data were corrected twice. Er was the ratio of the signal intensity of the enhancement peak to that of the intestinal wall before the start of enhancement, and each signal intensity was corrected at the same level.

### 2.6. Observation Indicators

Based on the postoperative pathological examination results, the accuracy of dark-lumen MRC examination results in the two groups was evaluated. ROC curve and ADC value were used as the criteria to evaluate the diagnostic efficacy of the two groups of methods for lesions, namely sensitivity and specificity. ME and Er were used to evaluate the lesion signal display effect of the two groups of MRC images.

### 2.7. Statistical Processing

Graphpad prism 5.0 software was used for statistical processing of each data. SPSS22.0 statistical software was used to compare the examination results of the two groups. Frequency (%) was used to represent the count data, and *χ*^2^ test was adopted to compare the differences. The measurement data were expressed as mean ± standard deviation, and the differences were compared by independent sample *t*-test. *P* < 0.05 indicated the difference in the index data between the two groups was statistically significant.

## 3. Results

### 3.1. Visual Assessment of Processed Images by Algorithm Group Compared with the Original Image and Convolutional Neural Network (CNN) Model Processing

The CNN model was selected as a reference. From subjective vision, the error of image was smaller and the accuracy was improved, especially the artifacts were removed and the image details were preserved, and the error was smaller, thus indicating that the algorithm group had higher image accuracy during reconstruction, and the observation and diagnosis of lesions were improved. The feature extraction image after the algorithm reconstruction showed that the pixel modulus difference of the algorithm group was weaker, reflecting that the imaging results were closer to the reference image (Figure 1, Figure 2, and Figure 3).

The sampling factor was 2.5–20 times. The three sampling trajectories were two-dimensional random sampling, Cartesian sampling, and phase coding sampling for K spatial data. Comparing the PSNR of the two algorithms in different iterations, it was observed that the algorithm group had higher signal-to-noise ratio on the reconstruction results, better retained the structural information of the image, and achieved higher resolution reconstruction (Figure 4).

### 3.2. Quality of Dark-Lumen MRC

Figure 5 showed the quality of dark-lumen MRC. The results showed that the images of rectum and sigmoid colon in the control group were better, which were 1.02 and 1.07, respectively. The images of descending colon and ascending colon were weaker, which were 1.33 and 1.51, respectively. The influencing factors of image quality were mainly due to respiratory motion artifacts, and there were wrap-around artifacts in the colon area. The ascending colon was close to the body's internal organs, which had the greatest impact and respiratory artifacts were heavier. The rectal image quality of the algorithm group was 0.31 higher than that of the control group. The sigmoid colon image quality of the algorithm group was 0.39 higher than that of the control group. The ascending colon image quality of the algorithm group was 0.15 higher than that of the control group. The cecum image quality of the algorithm group was 0.16 higher than that of the control group. The expansion of cecum and ascending colon was worse than that of rectum. The main reason may be related to intestinal stenosis and poor filling of proximal intestinal segments.

### 3.3. Comparison of the Results of Dark-Lumen MRC Examination in the Two Groups with the Results of Surgical Pathology and Infiltration Depth

The diagnosis of colon cancer was based on the staging criteria of Union for International Cancer Control (UICC). The number of cases in accordance with the imaging diagnosis of the two groups was illustrated in Figure 6. The number of correct cases in the algorithm group was 46, the number of diagnostic errors was 3 cases, and the accuracy was 93%. The number of correct cases in the control group was 41 cases, the number of diagnostic errors was 8 cases, and the accuracy was 83%. Compared with the accuracy, the algorithm group was 10% higher, indicating that the algorithm group had better diagnostic effect. The average infiltration depth of the algorithm group was 10.42, while that of the control group was 5.27, indicating that the algorithm group was more accurate in judging the infiltration depth (Figure 7).

### 3.4. Diagnostic Efficacy of Dark-Lumen MRC of Lesions in the Two Groups

ADC was 0.92 ± 0.14 mm^2^/s (min: 0.74, max: 1.30) in the control group and 1.55 ± 0.31 mm^2^/s (min: 1.22, max: 2.42) in the algorithm group. The ADC values of patients in the algorithm group were significantly higher than those of patients in the control group, with a statistically significant difference (*t* = 7.827, *P* *<* 0.001). The diagnostic efficacy of the two groups of lesions was evaluated using ROC curve and ADC values as criteria (Figure 8). The results showed that the area under the curve (AUC) = 0.992, *P* *<* 0.05, and when the critical threshold was taken as 1.25 mm^2^/s, the sensitivity of the diagnosis was 92.90% and the specificity was 94.70%.

### 3.5. Diagnostic Value of Dark-Lumen MRC for Colon Cancer

Colon cancer lesions showed homogeneous or heterogeneous significant enhancement, and the non-enhanced part showed high signal intensity in T2-HASTE. The comparison of ME and Er between the two groups was as follows: the comparison of ME values was 1.88 in the control group, 2.44 in the algorithm group, and the algorithm group was 0.56 higher. The comparison of Er values was 1.91 in the control group, 2.56 in the algorithm group, and the algorithm group was 0.65 higher (Figure 9).

## 4. Discussion

Colon cancer patients are increasing year by year, and young people have an increasing chance of colon cancer. Colon cancer is very common in clinical practice and usually occurs in the left colon, and local intestinal wall hypertrophy can indicate whether colon cancer occurs [10]. Surgical resection of patients with digestive organ cancer is a good treatment. Follow-up and observation should also be performed after resection to see whether there is recurrence. Early detection and timely surgical resection are the key to improve the clinical prognosis of patients. The proportion of long-term colon cancer in colorectal cancer is about 1%, and the proportion of deaths in patients with colon cancer is as high as 15%. Attention should be paid to clinical treatment [16]. For colon cancer, irregular obesity of the intestinal wall on all local or all imaging can be observed on the image. For different clinical drug therapies and treatment methods of these lesions, it is very important to select the appropriate examination method to identify these lesions [17]. Therefore, through the imaging examination of colon cancer, examination, and comprehensive analysis of clinical symptoms. The pathological finding on endoscopy of the large intestine is the decision on how to proceed with subsequent investigations for colon cancer. However, compared with imaging examination, biopsy has greater surgical risks and infection risks. Biopsy is only used when the condition is complex and difficult to examine. The condition of colon cancer is repeated and requires dynamic observation of changes in the patient's status at any time. Biopsy or endoscopy is invasive and not suitable for frequent use. It is a very large burden on the patient's heart and physiology [18]. Critically ill patients also need to confirm whether intestinal perforation and the cause of the disease, and the surgical conditions for colorectal endoscopy with worsening colon cancer are correspondingly complex and require specific sedatives and anesthetics when necessary [19]. Therefore, large intestine endoscopy has some limitations as a method for regular follow-up of colon cancer and long-term surveillance of colon cancer. The degree of intestinal lesions also requires observation of mucosal status, and colonoscopy cannot evaluate the depth and length of invasion as well as other complications of the colon, such as colitis [20].

At present, artificial intelligence algorithms are widely used in the field of medical image processing, for example, Li et al. (2021) [21] used deep learning models for the fusion processing of medical images and achieved excellent results in the diagnosis of diseases. Dark-lumen MRI based on artificial intelligence algorithm was used to diagnose colon cancer. The results showed that the image quality and diagnostic efficiency of the algorithm group were superior to those of the CNN algorithm treatment and the control group. The rectal and sigmoid images showed better quality, 1.02 and 1.07, respectively, and the descending colon and ascending colon images had weaker quality, 1.33 and 1.51, respectively. The influencing factors of image quality are mainly due to respiratory motion artifacts, there are wrap-around artifacts in the colon region, the ascending colon has the greatest effect due to its proximity to the organs in the body, the respiratory artifacts are serious, and the image quality of the cecum is 0.16 higher in the algorithm group than in the control group. Among them, the degree of dilatation of the cecum and ascending colon is worse than that of the rectal intestinal segment, and the main reason may be related to the stenosis of the intestinal lumen and the poor filling of the narrow proximal intestinal segment. The mean depth of invasion is 10.42 in the algorithm group and 5.27 in the control group, indicating that the algorithm group is more accurate in judging the depth of invasion.

## 5. Conclusion

It revealed that the diagnostic effect of dark-lumen MRI based on artificial intelligence algorithm was significant, ADC in the control group was 0.92 ± 0.14 mm^2^/s (min: 0.74, max: 1.30), ADC in the algorithm group was 1.55 ± 0.31 mm^2^/s (min: 1.22, max: 2.42). The ADC value of patients in algorithm group was significantly higher than that of patients in control group, with statistical difference (*t* = 7.827, *P* *<* 0.001). The correct number of cases was 46 and the diagnostic error number was 3 in algorithm group, with accuracy of 93%. The correct number of cases was 41 and the diagnostic error number was 8 in control group, with accuracy of 83%. In comparison, the correct rate was 10% higher in algorithm group than that in control group, indicating that the diagnostic effect was better in algorithm group. The mean value of invasion depth was 10.42 in the algorithm group and 5.27 in the control group, indicating that the algorithm group was more accurate in the judgment of invasion depth, had a good prospect of clinical application, and had guiding significance for the diagnosis of colon cancer.

## Figures and Tables

**Figure 1:** Visual assessment of processed images by algorithm group compared with the original image and CNN model processing. (a) Original image of colon cancer (b) colon cancer image processed by CNN model (c) colon cancer image processed by algorithm group.

**Figure 2:** Feature extraction lesion detection assessment after model processing. (a) Feature extraction lesion detection after CNN model processing (b) feature extraction lesion detection after algorithm group processing.

**Figure 3:** Comparison of PSNR values under two different sampling trajectories.

**Figure 4:** Comparison of PSNR between the two groups with 2.5–20 times sampling factor. *∗* represents statistical differences between groups.

**Figure 5:** Comparison of dark-lumen MRC imaging quality between the two groups. *∗* represents statistical differences between groups.

**Figure 6:** Comparison of correct and erroneous diagnosis cases between the two groups. *∗* represents statistical differences between groups.

**Figure 7:** Comparison of intestinal infiltration detection depth between two groups. *∗* indicates statistical differences between groups.

**Figure 8:** ROC curve of diagnostic efficacy of two groups of lesions.

**Figure 9:** Comparison of ME and Er values between the two groups. *∗* represents statistical differences between groups.

## Data Availability

The data used to support the findings of this study are available from the corresponding author upon request.
